# Efficacy and Safety of Temozolomide Combined with Radiotherapy in the Treatment of Malignant Glioma

**DOI:** 10.1155/2022/3477918

**Published:** 2022-02-15

**Authors:** Shoufeng Wei, Junde Li

**Affiliations:** ^1^Department of Neurosurgery, Zibo Central Hospital, Zibo 255000, Shandong, China; ^2^Department of Neurosurgery, Zibo Maternal and Child Health Care Hospital, Zibo 255100, Shandong, China

## Abstract

MG is a clinical common intracranial tumor, with the characteristics of strong invasion. In our study, we aim to explore the efficacy and safety of temozolomide combined with radiotherapy in the treatment of malignant glioma (MG) and its influence on postoperative complications and survival rate of patients. 120 MG patients admitted to our hospital (January 2019–January 2020) were chosen as the research objects and were randomly divided into group A (*n* = 60) and group B (*n* = 60). All patients were treated with radiotherapy, and patients in group A were additionally treated with temozolomide. The clinical efficacy, quality of life, incidence of adverse reactions, incidence of postoperative complications, survival rates, and average survival time of the two groups were compared. The objective remission rate (ORR), disease control rate (DCR), survival rates after one year and two years of follow-up, and the number of patients with improved quality of life in group A were markedly higher compared with group B (*P* < 0.05). The incidence of postoperative complications in group A was remarkably lower compared with group B (*P* < 0.05). The average survival time of group A was dramatically longer compared with group B (*P* < 0.001). There was no significant difference in the incidence of adverse reactions between the two groups (*P* > 0.05), and no new adverse reactions occurred in the patients. Temozolomide combined with radiotherapy can effectively improve the quality of life, treatment effect, and survival rate of MG patients, with a lower incidence of postoperative complications and better tolerance. Our finding indicates that temozolomide combined with radiotherapy has a high clinical application value. In addition, it indicates that this treatment method should be promoted in practice.

## 1. Introduction

Malignant glioma (MG) is a common clinical disease, with high malignant degree and strong invasive ability. The patients still face high risks of recurrence and death after surgical treatment, and their prognosis is poor [1–3]. In order to further improve the survival rate of patients, radiotherapy is often selected as an adjuvant therapy in clinical practice. However, radiotherapy cannot increase the tumor-free survival time of patients, and some patients still have a recurrence after radiotherapy, so radiotherapy alone has little effect [4–7]. In recent years, with the increasing attention to MG, some scholars have found that temozolomide can improve the overall efficacy of MG patients after radiotherapy. Temozolomide can penetrate the blood-brain barrier of patients and give full play to the role of alkylating agents, thereby reducing the possibility of recurrence. Moreover, patients will not have serious adverse reactions after taking it due to its mild toxicity, indicating that temozolomide has high clinical application value [8–11]. As we know, MG is a clinical common intracranial tumor, with the characteristics of strong invasion. Surgical treatment is often used in clinical practice, but patients still face a high risk of recurrence after surgery because it is difficult to completely remove lesions. Studies have shown that the postoperative survival time of MG patients is about one year, indicating that surgical treatment alone cannot improve the prognosis of patients. In current practice, radiotherapy is often used to prolong the survival time of patients, and alkylating agents are commonly used in radiotherapy, which can destroy the structure of MG cells. However, some tumor cells are not sensitive to radiotherapy. Long-term use of alkylation agents leads to adverse reactions such as bone marrow hematopoietic dysfunction, and patients are generally poorly tolerated. Thus, the application of radiotherapy is limited [12–14]. As people's awareness of MG continues to deepen, some scholars have found that temozolomide can improve the survival rate of MG patients, with high clinical application value.

Based on this, this paper analyzed the actual effect of temozolomide combined with radiotherapy in the treatment of MG, and 120 MG patients in our hospital were chosen for the research, with the summary report as follows.

## 2. Materials and Methods

### 2.1. General Data

120 MG patients admitted to our hospital (January 2019–January 2020) were chosen as the research objects and were randomly divided into group A (*n* = 60) and group B (*n* = 60). No statistical difference of general data was observed between the two groups (*P* > 0.05), as shown in Table 1. This study was approved by the hospital ethics committee.

### 2.2. Inclusion Criteria

The inclusion criteria of this study were as follows. (1) The patients or their family members were fully aware of the research process and signed informed consent. (2) The patients were diagnosed with malignant glioma by examination and had received surgical treatment [15, 16]. (3) The estimated survival time for patients was more than 3 months.

### 2.3. Exclusion Criteria

The exclusion criteria of this study were as follows: (1) the patients with mental problems or who were unable to communicate with others; (2) the patients with other organic diseases [17]; (3) the patients with infection symptoms [18].

### 2.4. Methods

All patients were treated with radiotherapy, with the specific steps as follows. (1) 6 MV external photon beam radiation was used in the radiotherapy by the conventional fractionated irradiation mode, with 2 Gy a day and 5 days a week. The treatment lasted for 2 months. (2) At first, the local large-field irradiation was used, and then the reduced-field high-dose irradiation was used when the irradiation dose reached 50 Gy. The total irradiation dose was 60 Gy.

The patients in group A were additionally treated with temozolomide, with the specific steps as follows. (1) Temozolomide (Jiangsu Tasly Diyi Pharmaceutical Co., Ltd.; NMPA approval no. H20040637) was taken orally at one hour before radiotherapy, and the dosage was 75 mg (m^2^ d) according to the height and weight. After starting the medication, routine examinations such as urine routine examination were conducted once a week, and liver and kidney function examinations were added at 3 weeks after starting the medication. (2) At one month after the end of radiotherapy, the patients were orally administered with 150 mg (m^2^ d) of temozolomide per day. After taking it for 5 days, the dose was increased to a maximum of 200 mg (m^2^ d) for a total of 150 days. (3) If the patients had adverse reactions during medication, the dosage should be adjusted.

### 2.5. Observation Criteria

1. Clinical efficacy: according to the World Health Organization (WHO) criteria of efficacy evaluation, the patients' condition was divided into complete remission (CR), partial remission (PR), stable disease (SD), and progressive disease (PD). CR + PR = objective remission rate (ORR). CR + PR + SD = disease control rate (DCR) [19].
2. Quality of life: the Karnofsky score was used to evaluate the quality of life of the two groups of patients. If the patients' Karnofsky scores increased by more than 10 points compared with those before treatment, it was an improved quality of life. If the patients' Karnofsky scores decreased by more than 10 points compared with those before treatment, it was a reduced quality of life. If the changing range of the patients' Karnofsky scores was between the above two, it was a stable quality of life [20].
3. Incidence of adverse reactions: adverse reactions included decreased white blood cell count, radioactive cerebral edema, nausea and vomiting, fever, myelosuppression, and anemia. The number of patients with adverse reactions in the two groups was counted [21].
4. Incidence of postoperative complications: postoperative complications included constipation, electrolytic disorder, pulmonary infection, consciousness disorder, upper gastrointestinal bleeding, and epilepsy. The number of patients with postoperative complications in the two groups was counted.
5. Survival rate: the survival rates of the two groups were compared after half a year, one year, and two years of follow-up.
6. Average survival time: the average survival time of the two groups was compared [22].

### 2.6. Statistical Treatment

In this study, the selected data processing software was SPSS 20.0, and the selected drawing software was GraphPad Prism 7 (GraphPad Software, San Diego, USA). This study included count data and measurement data, using *X*^2^ test and *T*-test methods. *P* < 0.05 indicated that the difference was statistically significant.

## 3. Results

### 3.1. Comparison of the Clinical Efficacy

The ORR and DCR in group A were obviously higher compared with group B (*P* < 0.05). See Table 2.

### 3.2. Comparison of the Quality of Life

The number of patients with improved quality of life in group A was obviously higher compared with group B (*P* < 0.05). See Figure 1.

### 3.3. Comparison of the Incidence of Adverse Reactions

There was no significant difference in the incidence of adverse reactions between the two groups (*P* > 0.05), and no new adverse reactions occurred in the patients. See Table 3.

### 3.4. Comparison of the Incidence of Postoperative Complications

The incidence of postoperative complications in group A was obviously lower compared with group B (*P* < 0.05). See Table 4.

### 3.5. Comparison of the Survival Rates

The survival rates after one year and two years of follow-up in group A were obviously higher compared with group B (*P* < 0.05). See Figure 2. By analyzing Figure 2, we can clearly see that, after six months of follow-up, there were 60 surviving patients (100.0%) in group A and 58 surviving patients (96.7%) in group B. The comparison showed *X*^2^ = 2.034 and *P*=0.154. After one year of follow-up, there were 54 surviving patients (90.0%) in group A and 44 surviving patients (73.3%) in group B. The comparison showed *X*^2^ = 5.566 and *P*=0.018. After two years of follow-up, there were 48 surviving patients (80.0%) in group A and 35 surviving patients (58.3%) in group B. The comparison showed *X*^2^ = 6.604 and *P*=0.010.

### 3.6. Comparison of the Average Survival Time

The average survival time of group A was obviously longer compared with group B (*P* < 0.001). From Figure 3, we can clearly see that the average survival time was 38.65 ± 6.24 months in group A and 25.11 ± 5.98 months in group B. The comparison showed *t* = 12.135 and *P* < 0.001.

## 4. Discussion

This study showed that the ORR and DCR in group A were markedly higher compared with group B (*P* < 0.05), indicating that taking temozolomide on the basis of radiotherapy could improve the overall efficacy. Temozolomide has high bioavailability and can be quickly absorbed by the body. It can penetrate the blood-brain barrier without being metabolized by the liver and give full play to the antitumor effect of alkylating agents. MG cells can increase to a certain amount in about 30 days due to the features of fast proliferation. In this study, the patients' medication time was more than 2 courses, with each course of 30 days, which was longer than one proliferation cycle of the tumor. The survival rates after one year and two years of follow-up in group A were remarkably higher compared with group B (*P* < 0.05), and the average survival time of group A was notably longer compared with group B (*P* < 0.001), indicating that temozolomide could effectively inhibit the proliferation of MG cells, reduce the speed of MG cell dissemination, and improve the prognosis of patients.

In addition, this study showed that there was no significant difference in the incidence of adverse reactions between the two groups (*P* > 0.05), and no new adverse reactions occurred in the patients. It indicated that the toxic reactions of temozolomide were mostly gastrointestinal reactions, and the symptoms were mild, which would not affect the patients' health. In general, temozolomide has fewer side effects and can be tolerated by patients during the medication period, with higher safety. In addition to the adverse reactions caused by radiotherapy, MG patients may also have a variety of postoperative complications such as epilepsy and electrolytic disorder, which are common in clinical practice. Without timely intervention, postoperative recovery process will be seriously hindered, and the efficacy will be affected accordingly [23, 24]. This study showed that the incidence of postoperative complications in group A was dramatically lower compared with group B (*P* < 0.05), indicating that patients in group A were in better physical condition after surgery. It is speculated that temozolomide can relieve the MG patients' clinical symptoms and enhance their body tolerance by controlling their disease condition. The patients' symptoms such as intracranial hypertension and epilepsy are relieved, so the incidence of complications is lower.

This study found that the number of patients with improved quality of life in group A was markedly higher compared with group B (*P* < 0.05), which was consistent with the research results of scholar Clara et al. In the study of Clara et al., the MG patients who had undergone surgery in the experimental group were treated with radiotherapy combined with temozolomide, while those in the control group were treated with radiotherapy alone. It was concluded that the Karnofsky score of the experimental group (83.21 ± 5.12 points) after 6 courses of treatment was dramatically higher than that before treatment and was higher than that of the control group (*P* < 0.001) [25], indicating that this combination therapy could improve the quality of life of patients, with better comprehensive effect.

## 5. Conclusion

In conclusion, temozolomide combined with radiotherapy can effectively improve the quality of life, treatment effect, and survival rate of malignant glioma patients, with lower incidence of postoperative complications and better tolerance. Our finding indicates that temozolomide combined with radiotherapy has a high clinical application value. However, our study still has some shortcomings. Our treatment method should be promoted in practice.

## Figures and Tables

**Figure 1:** Comparison of quality of life.

**Figure 2:** Comparison of survival rates. Note: the horizontal axis of Figure 2 from left to right represented half a year of follow-up, one year of follow-up, and two years of follow-up, and the vertical axis represented the number of surviving patients (cases). The line with dots represented group A, and the line with squares represented group (B). ^*∗*^indicated *P* < 0.05.

**Figure 3:** Comparison of average survival time ($\bar{x}\pm s$, months). Note: the horizontal axis of Figure 3 from left to right represented group A and group B, and the vertical axis represented the average survival time (months). ^*∗*^indicated *P* < 0.001.

**Table 1:** Comparison of general data.

Items	Group A (*n* = 60)	Group B (*n* = 60)	*X* ^2^/*t*	*P*
Gender			0.034	0.853
Male	35	34		
Female	25	26		
Average age (years old)	41.21 ± 6.20	41.23 ± 6.21	0.018	0.986
Karnofsky scores			0.069	0.793
≥80	51	52		
<80	9	8		
Tumor volume before surgery (m^3^)	6.54 ± 1.21	6.53 ± 1.23	0.045	0.964
Pathological grade			0.034	0.855
III	28	27		
IV	32	33		
Number of patients with residual tumor	38	39	0.036	0.849
Resection range			0.033	0.855
Residual tumor visible to the naked eye	30	31		
Total resection visible to the naked eye	30	29		
Tumor location			0.037	0.847
Subtentorial region	40	39		
Supratentorial region	20	21		

**Table 2:** Comparison of clinical efficacy (*n* (%)).

Items	CR	PR	SD	PD	ORR	DCR
Group A	24 (40.0)	24 (40.0)	6 (10.0)	6 (10.0)	48 (80.0)	54 (90.0)
Group B	12 (20.0)	20 (33.3)	12 (20.0)	16 (26.7)	32 (53.3)	44 (73.3)
*X* ^2^	5.714	0.574	2.353	5.566	9.600	5.566
*P*	0.017	0.449	0.125	0.018	0.002	0.018

**Table 3:** Comparison of the incidence of adverse reactions (*n* (%)).

Items	Decreased white blood cell count	Radioactive cerebral edema	Nausea and vomiting	Fever	Myelosuppression	Anemia
Group A	12 (20.0)	3 (5.0)	12 (20.0)	6 (10.0)	15 (25.0)	6 (10.0)
Group B	10 (16.7)	3 (5.0)	12 (20.0)	5 (8.3)	14 (23.3)	8 (13.3)
*X* ^2^	0.223	<0.001	<0.001	0.100	0.046	0.324
*P*	0.637	1.000	1.000	0.752	0.831	0.570

**Table 4:** Comparison of the incidence of postoperative complications (*n* (%)).

Items	Constipation	Electrolytic disorder	Pulmonary infection	Consciousness disorder	Upper gastrointestinal bleeding	Epilepsy
Group A	18 (30.0)	24 (40.0)	18 (30.0)	15 (25.0)	6 (10.0)	6 (10.0)
Group B	30 (50.0)	36 (60.0)	36 (60.0)	30 (50.0)	18 (30.0)	15 (25.0)
*X* ^2^	5.000	4.800	10.909	8.000	7.500	4.675
*P*	0.025	0.028	0.001	0.005	0.006	0.031

## Data Availability

The datasets used and/or analyzed during the current study are available from the corresponding author upon reasonable request.
